# Online Shopping Brand Sales Based on IoT Big Data Processing

**DOI:** 10.1155/2022/3833583

**Published:** 2022-03-26

**Authors:** Menglin Zhang, Xiaoyu Ma

**Affiliations:** ^1^Department of Fundamentals, Jiangsu Vocational College of Finance and Economics, Huaian 223003, Jiangsu, China; ^2^School of International Education, Jiangsu Maritime Institute, Nanjing 210000, Jiangsu, China

## Abstract

As a pair of closely related technical fields, “Internet of Things” and “big data” are gradually applied to the analysis of online shopping, which is very beneficial to promote the healthy and orderly development of the online shopping industry. This article uses the big data processing technology of the Internet of Things to analyze the influencing factors of online shopping brand sales based on the data collected by online questionnaires. It draws certain rules from it, and provides relevant marketing strategies for online shopping brand sales to assist its market positioning. According to the survey, the five aspects of online evaluation, brand awareness, online shopping community, online public opinion influence of related brands, and other brand information acquisition channels all have an impact on online brand sales. Especially women aged 25–35 will pay attention to online information, and 195 people will not choose to buy from brands with negative news. And during the purchase process, 186 people will check the online reviews of related brand products. Among them, there are 183 men aged 25–35 who will pay attention to online reviews.

## 1. Introduction 

According to CNNIC statistics, as of 2020, the number of search engine users reaches 790 million, and the utilization rate among netizens reaches 82.5%, as shown in Table 1. The popularity of the Internet has not only enabled people to share and obtain information, but also shaped a brand-new business model. Research shows that companies that choose e-commerce platforms for promotion account for the largest proportion, reaching 25.2%. Massive Internet search data records people's hobbies and needs, and provides a data foundation for social and economic development. Online shopping has become the mainstream mode of consumption in today's society. The selection of specific online marketing methods for small and medium-sized enterprises in 2020 is shown in Table 2.

1. Theoretical significance: through the search of relevant information, most of the research on online shopping uses statistical analysis methods and almost no one cares about the big data processing technology of the Internet of Things. This article discusses the influencing factors of online shopping brand sales through data preparation, Internet of Things big data processing technology, result analysis, discussion and induction. It provides a reference for the research of related online sales and e-commerce industry in the future.
2. Practical significance: this article collects relevant data through questionnaires, and uses the Internet of Things big data processing technology to analyze, so as to find some rules in online brand shopping. This provides marketing reference for companies engaged in online item sales and operations, and at the same time provides some theoretical foundations for the management of online platforms.

With the rapid development of the Internet of Things technology, many application fields related to the Internet of Things have emerged [1], such as GPS-based Internet of Vehicles systems, Internet of Things logistics systems based on RFID technology, as well as applications in the medical industry, and so on. However, relevant research and analysis on online shopping using the big data processing of the Internet of Things through the search of relevant information remain scarce. Therefore, this article will analyze the influencing factors of online shopping brand sales through the Internet of Things big data processing technology. It not only promotes the application research of the big data processing technology of the Internet of Things, but also provides certain market analysis value for the e-commerce field.

## 2. Related Work

With the advent of the Internet age, online shopping has become a mainstream shopping model. With the prosperity of the consumer market and the intensification of commodity competition, the producer-led marketing concept is clearly no longer in line with market rules, and more and more businesses are beginning to pay attention to consumers. Therefore, it is an opportunity to use the big data processing technology of the Internet of Things to analyze the influencing factors of online merchandise sales. Internet of Things (IoT) related applications have become an important area for engineers and researchers. Cai H provides a functional framework for identifying the acquisition, management, processing and mining of big data in the Internet of Things, and defines and describes several related technical modules based on their key characteristics and capabilities. He also analyzes the current research on the application of the Internet of Things and identifies the challenges and opportunities related to the research on the Internet of Things big data [2]. Big data refers to a collection of massive amounts of data that cannot be processed by traditional data processing tools and technologies. A large amount of climate data is collected from IoT weather sensor devices and NCEP. Manogaran G proposes a big data processing framework to integrate climate and health data to find the correlation between climate parameters and the incidence of dengue fever. The MapReduce framework based on In-Mapper is used to calculate the monthly average of the climate parameters for each latitude and longitude. Experimental results prove that, compared with the existing MapReduce algorithm, the In-Mapper based combiner algorithm has lower response time effectiveness [3]. The Internet of Things generates a lot of big data because it contains billions of devices connected to each other via the Internet. In order to process massive real-time geospatial big data, Limkar and Jha explores a scalable and efficient indexing method. A large number of experimental results show that the generated R-tree and its variants retain similar characteristics to the sequentially generated R-tree and its variants. This has excellent scalability, and reduces a lot of time to build indexes, index updates, and perform spatial range queries [4]. In recent years, e-commerce has been expanding at an alarming rate, and relevant Internet pages called e-services capes now occupy an important position in the business world. Therefore, Wu et al. conducts research on describing the nature of electronic service scenarios, and investigates the relationship between website credibility, website attitude, brand attitude, electronic word-of-mouth intention and purchase intention. A total of 290 responses are collected from Taiwanese consumers through online questionnaires. His research results show that the dimensions of the e-service landscape (aesthetic appeal, customization, usability, and financial security) have a significant impact on consumers' attitudes and trust in websites [5]. Ladhari et al. has also done related research. The goal of his research is to subdivide Gen female online shoppers based on their psychological, demographic and behavioral characteristics. The data comes from consumers of a female fashion retailer, and a total of 538 women shopping on this fashion retailer's website completed the survey. The results reveal four methods of online shopping: trend shopping, fun shopping, price shopping and brand shopping. It also identifies six shopping profiles, each with different goals: price shoppers, discovery shoppers, emotional shoppers, strategic shoppers, fashionistas and shopping fans [6]. In addition, Abbes I and others have studied to determine the stakes of the brand collaborative redistribution platform, and understand the influence of its internal and external characteristics on behavioral intentions. He also conducts a quantitative study on 214 people who had purchased second-hand goods online. The results show that the loyalty intention of the collaborative redistribution platform has an influence on the loyalty intention of the brand. The influence of platform service experience satisfaction on brand loyalty intention is mediated by platform loyalty intention [7]. Swapana and Padmavathy also conducts related research to study the relationship between the three dimensions of online second-hand shopping, customer satisfaction and repurchase intention. The responses received from 608 Indian online second-hand shoppers indicate that the dimensions of online second-hand shopping, such as price, website quality, nostalgia, and brand image, affect customer satisfaction. In addition, customer satisfaction has a positive impact on repurchase willingness. The research results show that online second-hand marketers enter emerging markets through effective online shopping strategies and provide intuitive guidance [8]. It can be seen that with the rise of online shopping, in the current era of large scale use of IoT big data to achieve efficient data processing, a decided lack of literature on the sales of online shopping brands remains. Therefore, in order to better analyze the influencing factors of online shopping brand sales, this article will use IoT big data processing technology. This has also promoted the further development of the Internet shopping era.

## 3. Internet of Things Big Data Processing Technology

Apriori algorithm and clustering algorithm are currently the two most widely used data mining algorithms [9, 10]. Its main research fields have a wide range of applications from pattern recognition to data analysis and image processing. Especially for the processing of big data in the Internet of Things, its characteristics are excellent, thus preferred by academic research and widely used in the industry [11, 12].

### 3.1. Clustering Algorithm

Two Step is a kind of clustering algorithm, which is used to solve the cluster analysis problem of massive data and complex category structure [13]. The difference between this algorithm and the traditional clustering algorithm is that the two types of clustering methods have small memory and fast calculation speed. Two-step clustering is to complete the clustering work through the two steps of preclustering and formal clustering [14, 15]. In the preclustering stage, data points in the dataset need to be inserted into the clustering feature tree (CF tree) one by one to realize the growth of CF tree. When the volume of the CF tree exceeds the set size, the CF tree needs to be thinned. On the contrary, the outliers of the thin CF tree are inserted into the CF tree. After reading all the data points, the potential outliers that cannot be inserted into the CF tree are the true outliers. Finally, the clustering features of the corresponding subclusters of the final CF leaf element are output to the next stage of the algorithm. As shown in from formulas (1) to (9) [16, 17].

(1) $$\begin{array}{c} {\overset{⟶}{\tilde{\Lambda }}}_{j}={\left({\tilde{\Lambda }}_{j1},\ldots ,{\tilde{\Lambda }}_{jD_{1}}\right)}^{T}={\left(\sum_{n=1}^{N_{j}}{\tilde{x}}_{jn1},\ldots ,\sum_{n=1}^{N_{j}}{\tilde{x}}_{jnD_{1}}\right)}^{T}, \end{array}$$

(2) $$\begin{array}{c} {\overset{⟶}{\tilde{\Sigma }}}_{j}={\left({\tilde{\Sigma }}_{j1},\ldots ,{\tilde{\Sigma }}_{jD_{1}}\right)}^{T}={\left(\sum_{n=1}^{N_{j}}{\tilde{x}}_{jn1}^{2},\ldots ,\sum_{n=1}^{N_{j}}{\tilde{x}}_{jnD_{1}}^{2}\right)}^{T}, \end{array}$$

where ${\overset{⟶}{\tilde{\Sigma }}}_{j}$ represents the linear summation of the attribute values of the data points in cluster *C*_*j*.

(3) $$\begin{array}{c} {\overset{⟶}{\ddot{N}}}_{j}={\left({\left({\overset{⟶}{\ddot{N}}}_{j1}\right)}^{T},\ldots ,{\left({\overset{⟶}{\ddot{N}}}_{jD_{2}}\right)}^{T}\right)}^{T}, \end{array}$$

where ${\overset{⟶}{\ddot{N}}}_{j}$ represents the sum of the squares of the attribute values of the data points in cluster *C*_*j*.

(4) $$\begin{array}{c} {\overset{⟶}{\text{CF}}}_{\langle j,j^{\prime }\rangle }=\langle N_{j}+N_{j^{\prime }},{\overset{⟶}{\tilde{\Lambda }}}_{j}+{\overset{⟶}{\tilde{\Lambda }}}_{j^{\prime }},{\overset{⟶}{\tilde{\Sigma }}}_{j}+{\overset{⟶}{\tilde{\Sigma }}}_{j^{\prime }},{\overset{⟶}{\ddot{N}}}_{j}+{\overset{⟶}{\ddot{N}}}_{j^{\prime }}\rangle , \end{array}$$

where ${\overset{⟶}{\text{CF}}}_{\langle j,j^{\prime }\rangle }$ represents clustering characteristics.

(5) $$\begin{array}{c} \zeta_{j}=-N_{j}\left(\frac{1}{2}\sum_{s=1}^{D_{1}}In\left({\hat{\sigma }}_{js}^{2}+{\hat{\sigma }}_{s}^{2}\right)+\sum_{t=1}^{D_{2}}{\hat{E}}_{jt}\right), \end{array}$$

where *ζ*_*j*_ represents the definition parameter of cluster *C*_*j*.

(6) $$\begin{array}{c} {\hat{\sigma }}_{js}^{2}=\frac{1}{N_{j}}\sum_{n=1}^{N_{j}}{\left({\tilde{x}}_{jns}-{\tilde{x}}_{js}\right)}^{2}, \end{array}$$

(7) $$\begin{array}{c} {\hat{\sigma }}_{js}^{2}=\frac{{\tilde{\Sigma }}_{js}}{N_{j}}-{\left(\frac{{\tilde{\Lambda }}_{js}}{N_{j}}\right)}^{2}, \end{array}$$

(8) $$\begin{array}{c} {\hat{\Sigma }}_{jt}=-\overset{\in_{t}}{\underset{k=1}{\sum }}\left(\frac{{\ddot{N}}_{jtk}}{N_{j}}In\frac{{\ddot{N}}_{jtk}}{N_{j}}\right)=-\frac{{\overset{⟶}{\ddot{N}}}_{jt}^{T}}{N_{j}}\cdot In\frac{{\overset{⟶}{\ddot{N}}}_{jt}}{N_{j}}-\left(1-\frac{{\overset{⟶}{1}}^{T}{\overset{⟶}{\ddot{N}}}_{jt}}{N_{j}}\right)\cdot In\left(1-\frac{{\overset{⟶}{1}}^{T}{\overset{⟶}{\ddot{N}}}_{jt}}{N_{j}}\right), \end{array}$$

(9) $$\begin{array}{c} d\left(C_{j},C_{j^{\prime }}\right)=\zeta_{j}+\zeta_{j^{\prime }}-\zeta_{\langle j,j^{\prime }\rangle }, \end{array}$$

where *d*(*C*_*j*_, *C*_*j*′_) represents the log-likelihood distance of cluster *C*_*j* and cluster *C*_{*j*′}.

The input of the clustering stage is the subclusters of the leaf element items of the final CF tree output by the preclustering stage. Therefore the work of this stage is to perform two-degree clustering on the subclusters according to the input data, and finally achieve the clustering results of the expected number of clusters. As shown in from formulas (10) to (17) [18, 19].

(10) $$\begin{array}{c} \text{BIC}\left(M_{i}\right)=-2Inf_{i}\left(x;{\hat{\theta }}_{i}\right)+k_{i}Inn, \end{array}$$

(11) $$\begin{array}{c} \text{BIC}\left(C_{J}\right)=-2L_{CJ}+KInN, \end{array}$$

(12) $$\begin{array}{c} L_{CJ}=\sum_{j=1}^{J}L_{Cj}=\sum_{j=1}^{J}\zeta_{j}, \end{array}$$

(13) $$\begin{array}{c} K=J\left(2D_{1}+\sum_{t=1}^{D_{2}}\left(\in_{t}-1\right)\right), \end{array}$$

(14) $$\begin{array}{c} \Delta_{\text{BIC}}\left(J\right)=\text{BIC}\left(C_{J}\right)-\text{BIC}\left(C_{J+1}\right),\;J=1,\ldots ,J_{0}, \end{array}$$

where Δ_*BIC*_(*J*) represents the difference between the BIC values of adjacent clusters.

(15) $$\begin{array}{c} r_{1}\left(J\right)=\frac{\Delta_{BIC}\left(J\right)}{\Delta_{BIC}\left(1\right)}, \end{array}$$

where *r*_1_(*J*) represents the rate of change of BIC value;

(16) $$\begin{array}{c} r_{2}\left(J\right)=\frac{d_{\min}\left(C_{J}\right)}{d_{\min}\left(C_{J+1}\right)},\;J=J_{I},\ldots ,2, \end{array}$$

where *r*_2_(*J*) represents the ratio of the closest cluster distance of clusters *C*_*J* and *C*_{*J*+1}.

(17) $$\begin{array}{c} J^{*}=\left\{\begin{array}{cc} J_{1},\text{if} & \frac{J1}{J}>1.15\\ \max\left\{J_{1},J_{2}\right\}, & \text{otherwise} \end{array}\right\}, \end{array}$$

where *J*^*∗*^ represents the best number of clusters selected from *J*_1 and *J*_2.

### 3.2. Apriori Algorithm

Apriori algorithm is a classic data mining algorithm for mining frequent itemsets and association rules [20]. The algorithm can not only discover frequent itemsets, but also mine association rules between items. It uses support and confidence to quantify frequent itemsets and association rules. The algorithm uses the prior properties of frequent itemsets to compress the search space. As shown in the following formula [21, 22].

(18) $$\begin{array}{c} \text{support}\left(A\Rightarrow B\right)=P\left(A\cup B\right), \end{array}$$

(19) $$\begin{array}{c} \text{confidence}\left(A\Rightarrow B\right)=P\left(B|A\right)=\frac{\text{support}\left(A\cup B\right)}{\text{support}\left(A\right)}, \end{array}$$

(20) $$\begin{array}{c} \text{confidence}\left(A\Rightarrow B\right)=\frac{\text{support}\_\text{count}\left(A\cup B\right)}{\text{support}\_\text{count}\left(A\right)}, \end{array}$$

where

 
support(*A*⇒*B*): it indicates the degree of support of the association rule
 
confidence(*A*⇒*B*): it represents the confidence level of the association rule

## 4. Application of Big Data Processing Technology in the Internet of Things

The actual practice of big data in the Internet of Things shows that reasonable systems and methods play a decisive role in the process [23]. The association rule in the Apriori algorithm refers to the common relationship between items, which is usually used to analyze sales. The Two Step algorithm supports numerical and subtype data. For large amounts of data, the calculation speed is faster and the execution efficiency is high. It provides great convenience in the application [24, 25], so this article will use the Internet of Things big data processing technology to study the influencing factors of online shopping brand sales.

### 4.1. Data Preparation

The survey method of this article is online questionnaire survey. It conducted 200 surveys on six groups of junior high school students, high school students, college students, young people aged 25–35, middle-aged people aged 35–50, and over 50 years old, and a total of nearly 200 questionnaire results for each group were recovered. At the same time, some face-to-face questionnaire surveys were conducted offline, and a total of 200 valid questionnaires were collected.

This article uses the Apriori algorithm and the two step algorithm to analyze the impact of online evaluation, brand awareness, online shopping community, related brand network public opinion influence, and other understanding channels on online brand sales, and conducts multiple fields. The results of this questionnaire survey are saved in an excel table, using its filtering function, selecting the T1 field (whether it will view and make relevant product reviews when shopping); selecting the T2 field (whether it will choose to buy products with high brand awareness); selecting the T3 field (whether it will buy through the online shopping community); selecting the T4 field (whether it will pay attention to and care about some negative news about the brand on the Internet) and selecting the T5 field (will it learn about the brand through other channels, such as the third website, offline word-of-mouth, etc.), and then filter out all records with a field value of “Yes”. The composition in Figure 1 sorts out five factors that affect online brand sales, including online evaluation and brand awareness, These five aspects are based on the sources that affect online brand sales, and it can be divided into three categories: one category comes from the consumer's online activity itself, that is, online evaluation; one category comes from online brands, including brand awareness of shopping websites, online shopping communities and related network information. Although these three elements will be controlled by the brand, the online activities of customers also play an important role; the last category comes from other channels, including third-party websites and offline word-of-mouth communication. The source of these two elements is not obvious, but they actually exist in the Internet. At the same time, these two elements are also mixed with a large number of online customer activities.

### 4.2. Data Analysis

The Internet continues to penetrate into the daily lives of netizens, and the number of online shopping users is increasing year by year. According to CNNIC statistics, as of 2020, the number of online shopping users in China has reached 989 million, and the Internet penetration rate has reached 70.4%. It is shown in Table 3. The development of commercial applications on the Internet is due to the rapid growth of the number of online shopping companies and that of Internet users who have begun to get used to this new way of online shopping. Therefore, this article will conduct a quantitative analysis of online shopping brand sales from the following five aspects.

#### 4.2.1. Online Evaluation

Online evaluation is a kind of online information, which mainly refers to the content itself spread by customers online. Every online behavior itself produces a large amount of information content, which will affect the popularity or reputation of online brands. Online information can often be analyzed from two aspects: information direction and information characteristics. Information direction refers to whether the information content itself has a positive or negative view of the online brand. Obviously, the direction of positive information can enhance the reputation of online brands, and vice versa, the direction of negative information will greatly damage the reputation of online brands. Information characteristics usually refer to the characteristics of the information, such as its manifestation, such as the length and type of the information, etc.; it also includes the inherent characteristics of the information, such as the credibility and legibility of the information. On the one hand, information characteristics will affect the information itself, and at the same time affect online brand sales through information.

As shown in Table 4, in November 2020, major apparel brands had a total of 730 online reviews by customers. Through analysis, PRADA pays more attention to online reviews of customers.

In the network context, the role played by the communicator and the receiver becomes difficult to distinguish, and the customer is both the communicator and the receiver. Generally speaking, the identity characteristics of the communicator and the receiver will obviously affect the credibility of the information they provide, thereby affecting the sales of online brands. The first is the professionalism of the two, which specifically refers to whether the communicator or receiver is an expert in this field. In the network environment, because the identities of the two are difficult to identify, false information is inevitable. But the professionalism can be judged from the content of the information it provides, such as customer reviews. It provides information in the form of reasoning, arranging knowledge, and discussing opinions, which obviously can be convincing. The second is the authority of the two. Compared with professionalism, authority is more difficult to identify. In traditional media, the authority is easy to judge, such as the authenticity and credibility of mainstream media reports. However, in the network environment, it is difficult to determine the authority due to the difficulty of identification. However, as some network applications begin real-name systems, the authority of the communicator or receiver becomes easier to judge. For example, the real-name authentication of Weibo, celebrity Weibo or expert Weibo is more authentic and credible due to its authority. Obviously, if online communicators and receivers are professional or authoritative, the information they provide is more likely to affect online brand sales. Therefore, the survey results based on online evaluation are shown in.

The results of the male and female role survey also showed that, when most people shop, they check reviews and make comments on related product, as shown in Figure 2, the highest enthusiasm for the activity was women aged 25–35, with 186 people. Followed by female college students and 25–35-year-old males, 183 people, and 172 male college students will also have this activity. This shows that most people agree that online reviews have a great influence on their brand choice.

#### 4.2.2. Brand Awareness

This article believes that brand awareness also occupies an important position, and its influence on online brand sales is second only to online customer reviews. Compared with offline shopping, online shopping has its own uniqueness, so many people pay more attention to the brand when buying things. The inability of consumers to directly touch and feel the product increases the difficulty of product quality judgment. It can be seen from this that in the highly competitive e-commerce market, brand awareness is the standard by which buyers' measure stores. The higher the popularity of the store, the natural flow of people will increase, and the sales will also increase. The result of the influence of brand awareness on brand sales is shown in Figure 3.

As mentioned above, brand awareness accounts for a large proportion of online brand sales. 132 male college students and 161 25–35-year-old males will choose well-known brands when shopping, and agree that the brand's products have certain quality assurance. As shown in Figure 3, female college students and women over the age of 25 trust the quality of well-known brands, and their numbers are above 110. This shows that brand awareness has a great influence on sales.

#### 4.2.3. Online Shopping Community

Online shopping community generally refers to a special discussion space built by merchants in order to activate the atmosphere of online shopping and enhance the initiative and enthusiasm of customers in online activities. Customers share shopping in the community, post orders and post product or service reviews. In the purchase process, users click on the product information of interest according to their own needs, and these evaluations can increase the attention of other customers to the product, thereby prompting customers to click and browse the product information. The results of the face-to-face questionnaire survey in this article show that 30.27%, 22.51%, and 17.25% of users agree that they will click on product information with higher attention, as shown in Figure 4. Not only that, the community homepage has a search function, which can help customers find their ideal products quickly and easily. It can be seen that the huge online activities in the online shopping community will undoubtedly involve all aspects of online brand sales. Therefore, this kind of combined customer online activities dominate online brand sales.

It can be said that the online shopping community is the essence of customer online activities. A variety of customer online activities gather in the online shopping community, such as the communication between the brand and the members, and that between community members. Relying on the contributions of relevant parties, these activities themselves have been continuously optimized. The information provided by community interaction is more comprehensive and specific, which can be said to be the essence of customer online activities. At the same time, the online shopping community itself has a judging function. For example, posts that are popular with customers tend to have a higher click-on rate, more information value, and more active participation among netizens. The refined customer online activities are more credible. Thus both the brand and the customers themselves are making contributions to customer online activities. For example, sellers will show better-selling products through online communities, while buyers will help latecomers through their own shopping experience. Of course, the information will undoubtedly improve the authority and professionalism of customers' online activities. This kind of information content through the discussion can summarize the whole picture of the problem better, thus making the customer's online activities more authentic and credible. Such authentic online activities will undoubtedly affect the sales of online brands. The results of the online shopping community's influence on brand sales are shown in Figure 5.

As shown in Figure 5, many young people are very active in online communities.

Regardless of gender, groups from junior high school students to 25–35 young people believe in product reviews in online communities. The number of them is more than 100, and the highest number is 25–35 year-old women, reaching 153. This shows that the marketing of online shopping communities has a positive role in promoting online brand sales.

#### 4.2.4. Network Message

With the rise of the Internet, there is a huge amount of information on the Internet. In order to get more display opportunities for information, or to allow online brands themselves to gain more public opinion support, brands will inevitably hire network naval forces to spread information, thus creating a false scenario. Network naval forces belong to a relatively special group in the Internet. Generally speaking, the network navy is employed by the brand side, and its behavior is mostly controlled by the online brand side. In addition to the normal way of brand communication, the current online brand communication also has to rely on a large number of network navigators.

First of all, network naval forces generally disseminate information on a large scale, which greatly enriches online information. Although the quality of information varies from good to bad, it often has an absolute advantage in quantity. In terms of the nature of online information provided by the network navy, there are currently two main types: positive online information and negative online information. Positive online information is mostly to promote the enthusiasm of the brand itself or the product, thereby enhancing the popularity and reputation of the online brand. Negative online information is generally done by competitors, who use the network navy to publish information that is unfavorable to the brand itself or the product, and at the same time use malicious posts to attract the public's attention and combat competitors. It is not difficult to see from the above that a large amount of information created by the network navy makes people difficult to distinguish between true and false, and this online information will also affect people's evaluation of the brand.

Secondly, the network navy's all-round online promotion behavior. The promotion behavior of the network navy is often planned and implemented by the public relations company for three-dimensional promotion. There are five common situations in the online promotion of network navy: First, community promotion. It provides dissemination services in communities and forums. Relying on the requirements of the brand or related parties to formulate forum or community communication strategies and specific implementation rules, while targeting target consumers, implement forum precision marketing, and follow up services in accordance with the marketing plan. Second, hot speculation. It uses the focus of attention of the public, media, and netizens to follow up, and creates high-relevant communication topics, and controls and guides them in this process. Third, event marketing. It manufactures hot events related to online brands, carries out all-round packaging and hype, attracts the attention of relevant parties, and at the same time attracts follow-up reports from the media to a certain extent, extends the influence of communication, in order to achieve the goal of online brand marketing. For example, the event marketing of Ganlu has become the target of media hype to a certain extent. Fourth, Weibo and blog marketing. It uses Weibo, blogs, etc. To spread products or brands. There are mainly the following three forms: well-known blog marketing, self-built blog marketing and group-built blog marketing. These three forms are usually implemented in combination. Fifth, deleting negative news. It contacts search engines, uses artificial means or a combination of other illegal means to instantly obtain negative information related to online brands in the Internet space, and guide or clear it, especially suitable for active defense or prevention of brands negative information. From the above, the online promotion of the network navy has a guiding effect on the network information of related brands, thereby affecting the sales of online brands. Therefore, this article conducted a survey based on the elements of network information, and the survey results are shown in Figure 6.

In the Internet age, people can learn all kinds of information quickly without using traditional media, which brings great convenience to people. Therefore, the brand side will also hire the network navy to create the network focus, attract people's attention, so as to enhance the awareness and reputation of its own brand. As shown in Figure 6, women aged 25–35 will pay attention to online information, but for brands with negative news, they will not choose to buy, and the number of women reaches 195. Similarly, 182 men aged 25–35 also agreed with this view, and 186 female college students also expressed support. This shows that the orientation of positive online news has a certain boosting effect on brand sales.

#### 4.2.5. Other Channels

Analysis of elements based on other channels, including third-party platforms, offline word-of-mouth communication.

*(1) Third-Party Platform*. Third-party platforms refer to customer online activities that appear on other Internet platforms in addition to the brand's own online marketing channels. Third-party websites also gather a large number of customer online activities. Since customer online activities appear on third-party platforms, its authenticity is stronger, and it is easier to get customers' affirmation.

First, the online activities of customers on third-party platforms are displayed. The ways for customers to display their activities online on third-party platforms are mainly self-media such as communities, forums, blogs, Weibo, and WeChat. After general customers purchase behaviors, they will evaluate their satisfaction with the products, and the customers will display information about the products in the relevant media or describe their own shopping experience. This kind of display activity that occurs on the self-media is generally consumer spontaneous. Therefore, relatively speaking, it is more authentic and credible. Of course, it is also possible for businesses to hire network naval forces to engage in display activities.

Second, the spread of customer online activities on third-party platforms. The proliferation of customer online activities on third-party platforms is reflected in the uncertainty of the space for online activities. It can be said that on the entire Internet platform, customer online activities can exist. The Internet is a “global village,” so customer online activities can theoretically spread arbitrarily on the Internet platform. At the same time, different consumers have different interests and hobbies, and the space of online activities diffusion generally conforms to the interests of customers. Because different consumers browse different platforms, the diffusion of customers' online activities has a strong uncertainty. Of course, due to its relative independence, customer online activities appearing on third-party platforms are essentially not under the control of brand marketing, but are also the self-expression of customers themselves. Therefore, in addition to the marketing of the network navy, the authenticity of the information on the third-party platform is relatively high. For example, customers often browse other platforms to learn about them when shopping, or use search engines to view online activities such as related product information of other brands. This article is drawn through a face-to-face questionnaire survey, as shown in Figure 7. 31.6%, 23.85% and 18.56% of its users agree that they will search for product information or product reviews on the Internet. This shows that their purchasing decisions are largely influenced by the information on these third-party platforms. These online activities can reflect the value of customer online activities on third-party platforms. Therefore, online activities on third-party platforms also have an important impact on online brand sales.

*(2) Offline Word of Mouth*. In addition to third-party platforms, offline word-of-mouth communication from customers outside the Internet will also affect online brand sales. Of course, because the research perspective of this article is based on the Internet, the article only discusses some offline word-of-mouth activities related to online brands and their impact on online activities. Most customers will comment on this purchase after their online brand buying behavior occurs. Except for the evaluations on the Internet platform, this article believes that most of the customer's evaluations after shopping will be spread offline. This study also found through face-to-face questionnaire surveys that, in addition to online search, introductions by relatives and friends are also an important channel for customers to obtain product or service information. As shown in Figure 8, its proportion is as high as 29.87%.

Obviously, this kind of communication spreads the influence of online brands beyond the Internet, and has a significant impact on online brand sales. For example, after customers purchase a certain brand of goods online, they will spread word of mouth on real social relationships, such as relatives and friends. Of course, most of this kind of word-of-mouth communication obviously appears outside the Internet platform, which has a significant effect on attracting potential target consumers. If this word-of-mouth communication is positive, it will encourage more customers to buy a certain brand online. Conversely, negative offline word-of-mouth will affect online brand reputation.

If potential customers are attracted by offline word-of-mouth communication and enter the Internet space, the role of offline word-of-mouth communication has become prominent. And new potential customers often have the following two online behaviors:

  The first is to seek online word of mouth.
  Because the customer obtains the relevant information of the brand offline, the information about the brand has a high degree of uncertainty, and the customer is eager to seek more information to eliminate this uncertainty. Therefore, online activities for seeking brand reputation have emerged. Customers can obtain more relevant information by searching, posting, consulting and other means. Therefore, this kind of customer activity itself promotes the enrichment of online information resources, and can provide relevant information content to latecomers.
  The second is to verify offline word-of-mouth behavior.
  It is not difficult to see that on the one hand, customers search for online word-of-mouth information through various online methods, and on the other hand, customers will also verify offline word-of-mouth behavior. Because customers cannot be sure of the authenticity of the information provided by offline word-of-mouth, the process of seeking information is also a process of verification. If online word-of-mouth and offline word-of-mouth match, then the customer's brand impression will deepen, thereby forming trust in the brand. On the contrary, if the information that the customer seeks on the Internet platform does not match the information received offline, then the customer's sense of distrust will increase, which will affect the evaluation of the brand. In summary, whether it is seeking online word-of-mouth behavior or verifying offline word-of-mouth behavior, the customer's activity itself has already constituted an impact on online brand sales. The results of the survey are shown in Figure 9.

The advent of the information age has made it easy for people to obtain various information resources. The survey shows that the majority of people obtain online brand-related information through other channels. As shown in Figure 9, men and women aged 25–35 will search for third-party platforms to learn relevant online brand information, and the number of them is more than 180. People aged 35–50, especially those over 50, prefer to obtain relevant brand product information through recommendations from relatives and friends, and the number of them is more than 130.

It can be seen that the influence of online brand sales comes from five aspects. The article only summarizes the five main factors that affect online brand sales. In the actual Internet environment, there may be other online activities that affect online brand sales. This article can only provide important influencing factors, and cannot completely describe all the influencing factors of online brand sales. In addition, the five aspects will interact and influence each other internally.

### 4.3. Suggestions on Online Brand Marketing Strategies

As mentioned above, the five factors of online evaluation, brand awareness, online shopping community, online news, and other channels affect online brand sales. Accordingly, this article summarizes the impact of five factors on online brand sales and give some marketing suggestions, which are mainly reflected in the following aspects:

First, it enriches potential online information resources.

In the era of new media, information about related products or services can be gathered together through hyperlinks and other means, so that users can obtain massive amounts of information about products or services. If a user finds an advertisement for a certain product or service on the Internet, he will use various Internet tools to understand the product. If the product does not have complete information, customers can search for it online. Therefore, from the perspective of online information content, potential online information resources will continue to be enriched due to the continuous contributions of customers. At the same time, a large number of customer online activities are gathered together in the form of keywords, providing customers with complete online information resources through hyperlinks. Therefore, based on the massive information of Internet products and the means of hyperlinks, customers can learn about all product systems from individual product information, as well as information about products and related brands. Therefore, in the era of new media, with the continuous integration of information, the content of online information resources has been greatly enriched. This has increased online brand sales to a certain extent.

Second, the promotion of online channels.

In the era of traditional media, the interaction between customers and businesses is extremely restricted due to the long time for feedback and limited feedback channels. For example, advertisement information in newspapers cannot provide timely feedback on the product. Even after the feedback, the time for the company to receive the feedback information is very long. Therefore, it is very important to make full use of various feedback channels in the new media era to interact with online customers in an integrated way. With the development of Internet technology, there are more and more ways to conduct product promotion online. For example, after consumers see relevant product information on the Internet, they can immediately click on the product's website or link to view it. At the same time, they will spread relevant product or brand information in real time through various media around them. In the current era of increasingly rich media methods, interactivity has become one of the prominent signs of communication between customers and brands. With the development and popularization of various applications on the Internet, the online activities of customers on various applications are interactive, multi-directional, and participatory, which greatly promotes the promotion of online brands or products. Therefore, the upgrading of online promotion channels is indispensable, such as blog promotion, WeChat promotion, and various application software promotion.

Third, offline word-of-mouth and online word-of-mouth are combined.

In addition to its own online promotion of brand reputation, customers also play a decisive role in the spread of brand reputation. Therefore, it is necessary to combine offline word-of-mouth with online word-of-mouth.

#### 4.3.1. Offline Reputation of Online Brands

The offline reputation of a brand is formed through communication between people. In daily life, customers obtain online promotion information of related brands by communicating with people around them. Out of trust in people around them, they are more convinced of the authenticity and reliability of related brands. Each customer is actually playing the dual role of information disseminator and information receiver. The information that customers get about online brands is more likely to be the experience dissemination of the information disseminator through the experience of purchasing the online brand in person, or it may be the information about the online brand that the information disseminator obtains from other customers. Although there are differences in the personal needs of each customer, this has also prompted customers to recognize the quality of related brands more. The spread of online brands by customers offline has gradually formed the offline reputation of online brands.

#### 4.3.2. Online Reputation of Online Brands

The online reputation of online brands is mainly formed through online customer reviews. In the era of information sharing, after customers purchase related branded goods online, online platforms can make text comments on related branded goods or services, making relevant information about online brands more intuitive and transparent. Among these reviews, there are not only reviews of related brand products, but also those of shopping platforms, and there are both positive and negative reviews. The spread of these comments through the Internet has gradually formed the online reputation of online brands.

#### 4.3.3. Combining Offline Word-of-Mouth with Online Word-of-Mouth

From the perspective of online brand communication, the development of a brand cannot rely on online or offline unilateral communication. Therefore, the word-of-mouth of an online brand needs to be formed by the combination of online and offline. Customers make reviews when doing purchases, and brands can continuously improve their services based on customer reviews to further meet customer needs. This shows that customers play a leading role in the formation and development of online brands.

Fourth, the communication of the online brand itself is combined with that of customers.

From the perspective of communication, customers are both consumers and communicators. Therefore, the combination of online branding and customer communication will generate a better effect. For example, when customers search for relevant brand product information, they will communicate with brand staff in a timely manner to obtain the information they want. Of course, customers can also consult various experts through various communities and forums, and all this information can only be obtained by searching for them. The propagation process is shown in Figure 10. At the same time, on the Internet platform, all consumer information can be disseminated a second time, and customers can forward it through various platforms such as Weibo, WeChat, and communities. For example, through various self-media means, customers can forward the information content of their favorite products or services to relevant people or recommend them to other friends. This kind of dissemination that customers actively forward will make the secondary dissemination wider to a certain extent. Therefore, customer communication is as important as the brand's own communication, which requires special attention.

Fifth, customers collaborate to participate in online brand communication.

Online brand communication activities require the active participation of customers, so the brand needs to mobilize the enthusiasm and enthusiasm of customers. At the same time, it is also necessary to strengthen the interaction with customers, so as to provide useful information to the brand during the interaction process in order to better carry out brand communication activities. For example, A is a popular search client. When general consumers do not understand brand information, they can search for answers to related brand information through A, and A generally has similar questions or answers from previous consumers, which can meet the needs of consumers. Of course, customers can also open an account A to provide their views on the brand, and it is precisely because of this that makes A's information more comprehensive and true, and provides more comprehensive information for future customers. It can be seen that the collaborative participation of customers in online brand communication has become a norm on the Internet, and the process of participation is also the process of brand information integration. Online brands can also extract the essence of relevant information. Customers can feed back good products or services to the brand, so that relevant brand information can be better displayed to customers, thereby increasing the credibility and promotion of the brand.

## 5. Discussion

This article conducted 200 effective online questionnaires for six groups of college students and young people aged 25–35 to collect relevant data to analyze the influencing factors of online shopping brand sales. The main findings of this article are analyzed as follows:

1. Online evaluation. More than 180 men and women aged 25–35 said that they would pay attention to the evaluation of related brand products when shopping;
2. Brand awareness. Young people aged 25–35 will pay more attention to brand awareness, and college students also express that they prefer branded products with brand awareness, and the number of them is more than 110. Compared with women, men will recognize the quality of branded goods better, and the number of men from college students to men over 50 years old is more than 110;
3. Online shopping community. The survey results in this article show that young people are more active and proactive in participating in the community. People after 35 years old, because of different interests and low mobile phone usage, platforms such as communities are not the main channels for understanding product information;
4. Network information. In the era of information sharing, adults will quickly learn about online news through platforms such as TV and have corresponding likes and dislikes. Therefore, online brands need to actively guide the brand's correct and true online news to increase the credibility of the brand to customers.
5. Channels to learn about other brand products. It mainly focuses on the two aspects of third-party platforms and offline word-of-mouth communication. The 25–35-year-old youth association learns about relevant brand information through the third online platform, and the number of them is more than 180. The majority of men and women aged over 35 learn about relevant product information through the introduction of relatives and friends, and the number is more than 170.

It is not difficult to see that five aspects, including online evaluation and brand awareness, all affect online brand sales.

## 6. Conclusion and Outlook

Based on the big data processing technology of the Internet of Things, this paper analyzes the influencing factors of online shopping brand sales. It conducts an online questionnaire survey of people from junior high school to over 50 years old. According to the survey, the five aspects of online evaluation, brand awareness, online shopping community, related brand network news, and other brand product information acquisition channels all affect online brand sales. This article puts forward some marketing strategies in a targeted manner. First, by enriching online resources, customers can retrieve and consult relevant brand product information and learn about related services through major platforms. Second, through online promotion, customers can see brand product information on their frequently active platform, and can learn product information by clicking on the link to complete the purchase behavior. Third, through the combination of online and offline to spread brand reputation, customers will share and evaluate on third-party platforms after purchase, and the brand can make corresponding adjustments based on customer reviews to further meet the needs of the market. Fourth, in addition to self-dissemination, we should also pay attention to customer communication. Brand staff can conduct publicity based on answering customer questions, and customers will disseminate relevant information on other Internet platforms. In this way, the promotion of the brand has been further increased. Finally, customers collaborate to participate in online brand communication. Online brands can mobilize the enthusiasm of customers, better promote the brand by understanding customer needs, and increase the credibility of the brand.

The article uses a questionnaire to quantitatively analyze the sales of online shopping brands based on the big data processing of the Internet of Things, but there are still many shortcomings. First, the depth of the article research is not enough, only five aspects of online evaluation, brand awareness, etc. Have been investigated and researched, and no more in-depth research has been conducted on a certain factor; second, the data of the article also has its shortcomings. There are many factors that affect online brand sales. The survey sample only selected five aspects as research data, such as consumer psychology, consumer care elements, and so on. These two aspects are the follow-up work of this article.

## Figures and Tables

**Figure 1:** Based on the five aspects of the impact of online shopping brand sales composition.

**Figure 2:** Online evaluation survey results. (a) Male survey results on online evaluation. (b) Women's survey results on online reviews.

**Figure 3:** Survey results of brand awareness. (a) Men's survey results on brand awareness. (b) Women's survey results on brand awareness.

**Figure 4:** Product information or evaluations with a high degree of attention.

**Figure 5:** Survey results of online shopping communities (a) Male survey results on online shopping communities (b) Women's survey results of online shopping communities.

**Figure 6:** Survey results of network information (a) Men's survey results on Internet information. (b) Women's survey results on online information.

**Figure 7:** Histogram of product information searched by third-party platforms or search engines.

**Figure 8:** Column chart of channels for online shopping groups to obtain information on goods or services.

**Figure 9:** Survey results from other channels (a) Men's survey results on other channels (b) Women's survey results of other channels.

**Figure 10:** Online communication process.

**Table 1:** Use of search engines by Chinese netizens.

Years	Data	
	Chinese search engine user scale/ten thousand people	Utilization rate among netizens (%)
2017	63956	82.8
2018	68132	82.2
2019	72106	81.8
2020	79461	82.5

**Table 2:** Selection of specific online marketing methods for SMEs in 2020.

Corporate internet marketing	The proportion (%)
E-commerce platform promotion	25.2
E-mail marketing	23.5
Search keyword ads	15.3
Internet brand advertising	13.2
Online video advertising	9.3
Network soft article	8.7
Search engine optimization	2.5
Network alliance, joint marketing	2.3
Other online marketing activities	1.1

**Table 3:** Statistical data table of Chinese internet development status.

Years	Data	
	Number of online shopping users	Internet penetration rate (%)
2017	7.72	55.8
2018	8.28	59.6
2019	9.03	64.5
2020	9.89	70.4

**Table 4:** Customer online evaluation questionnaire of major clothing brands in November.

Clothing brand	Evaluation attributes		
	Praise	Average	Negative ratings
PRADA	425	29	3
ONLY	46	16	0
ZARA	52	18	16
HM	103	12	10

## Data Availability

All the data used are included in the article.
